The article "Design of Sports Training Simulation System for Children Based on Improved Deep Neural Network" was retracted in 2023. Reasons: signs of a paper mill; suspected computer-generated content; unreliable results or conclusions; concerns about the data.

# Design of Sports Training Simulation System for Children Based on Improved Deep Neural Network

**DOI:** 10.1155/2022/9727415

**Published:** 2022-05-31

**Authors:** Xuesheng Wang, Qiuhong Han, Feng Gao

**Affiliations:** ^1^Institute of Physical Education, Huzhou University, Huzhou, Zhejiang 313000, China; ^2^Jiaxing College Sports and Military Training Department, Jiaxing University, Jiaxing, Zhejiang 314000, China

## Abstract

With the development of AI technology, human-computer interaction technology is no longer the traditional mouse and keyboard interaction. AI and VR have been widely used in early childhood education. In the process of the slow development and application of voice interaction, visual interaction, action interaction, and other technologies, multimodal interaction technology system has become a research hotspot. In this paper, dynamic image capture and recognition technology is integrated into early childhood physical education for intelligent interaction. According to the basic movement process and final node matching in children's sports training to judge children's physical behavior ability, attention is paid to identify the accuracy and safety of movement. The input images and questions are from the abstract clipart dataset of dynamic image recognition and the self-made 3D dataset of Web3D dynamic motion scene with the same style, which is similar to the action content in the actual preschool training teaching. Therefore, according to the idea of process capture and target recognition, on the basis of the original conditions of the recognition model, a new recognition model is developed through Zheng's target detector. The modified model is characterized by higher accuracy. Weapons need to combine process recognition and result recognition. The experimental results show that the improved model has the obvious advantages of high precision and fast speed, which provides a new research idea for the development of children's physical training simulation.

## 1. Introduction

The development of children's sports is not only the evidence of the development of China's sports cause but also the foundation of the construction of sports power. Children involved in sports, because there is no systematic learning, may not be able to improve the technical level due to the nonstandard movement or even have sports injuries [1]. Therefore, children's movements need to be reviewed and improved frequently. Traditional training methods need professional sports coaches for one-to-one teaching, there are high labor costs and low flexibility problems, and how to carry out children's sports teaching and training through a more simple and effective way is an urgent problem to be solved [2].

Computer-assisted instruction (CAI) is a teaching method that uses computers to communicate teaching materials and evaluate learning effects (Suleman et al.) [3]. In order to improve students' learning interest, learning ability, and academic performance, the media such as image, text, sound, and video can be mixed in the teaching process. CAI software can actually refer to any type of computer applications in the teaching process, including drills and practice, simulation, teaching exercises, supplementary exercises, teaching management, database development, programming, and other applications with different functions.

The research and application of computer-aided instruction technology has been making progress in the continuous exploration of researchers. Bartholomew et al. found that interactive multimedia computer games can promote students' self-management ability [4]. Bernard et al. found that computer-aided instruction software can help autistic children learn problem-solving strategies to a certain extent [5]. Sângeorzan et al. developed a computer-aided teaching system that can simulate stack changes in the process of code compilation and generation by using FLASH and found that teaching efficiency was effectively improved by using this system [6]. Through these application examples of computer-aided instruction technology, we can see that computer-aided instruction has played an important role in many aspects. Suleman et al. proved that CAI has a significantly positive impact on students' academic performance and knowledge memory [3]. Through the experiments and conclusions of the above researchers, it can be seen that the use of computer teaching as auxiliary on the basis of traditional teaching has a positive effect on the improvement of students' academic performance.

The purpose of this paper is to create an intelligent interactive framework in the Web3D environment, so that children can have an immersive interactive experience in physical education class and, at the same time, add visual technology in artificial intelligence learning to the virtual screen. The system can evaluate whether the athletes can accurately make the actions in the screen. In addition, another significance of this paper is based on the perspective of deep learning of motion simulation system. Most of the motion simulation systems only focus on improving the accuracy of motion and only make innovations in algorithms or software in computers. However, in order to provide actual interactive services to users, a physical interaction platform is required. Therefore, this paper introduces the new application and value of visual question answering technology by developing a virtual education platform for intelligent interaction with users. It provides a new idea for the development of sports assistance system and is of great significance for the promotion of sports projects.

## 2. Improved Deep Neural Network Algorithm Theory

Artificial Neural Network (ANN), referred to as neural network (NN), is a distributed parallel information processing algorithm model that imitates the neural behavioral characteristics of biological brain. Neural network achieves the purpose of information processing by adjusting the complexity of the interconnected relations between a large number of nodes in the system [7], through the design of the corresponding algorithm, to simulate the related intelligent activities of the human brain, so that the computer can technically achieve the same ability as human beings to deal with related problems.

### 2.1. Traditional Artificial Neural Network

The traditional Artificial Neural Network has been studied by human beings for a long time [8]. In interdisciplinary and large-scale studies, the study of neural networks has occupied a place. The natural responses of biological nervous systems to the real world can be modeled by the structure of neural networks. In the research field of artificial intelligence deep learning, neural network also refers to neural network learning. The smallest unit of the neural network is the neuron, which is similar to the biological nervous system and is also interconnected among neurons [9]. In the case of neurons by external stimuli, nearby neurons can receive the excitement of transfer to the corresponding chemical; nearby neurons state has produced a change in potential; when the potential of a neuron is more than a certain critical value, the neurons are activated; at the same time, the neurons continue to send related chemicals to the neighboring neurons.  Figure 1 of neuron is as follows:

In the neuron model, when other neurons begin to transmit some weighted signals to the current neuron, the current neuron will compare its critical value with the relevant signals received and then transmit the signals to the next neuron after processing the activation function. Neural networks are networks that are connected in a particular way like this [10]. It is still not clear whether the current structure of neural network mathematically simulates the nervous system of the organism. At the beginning, neural network is just a simple model integrating multiple linear functions. Data and problems in real life are usually much more complex and often not linearly separable. The emergence of activation function introduces nonlinear factors into neural network and makes neural network able to approach any nonlinear function arbitrarily, which can be applied to many nonlinear models and solve more and more complex problems.

Common activation functions are Sigmoid function, Tanh function, ReLU function, and some improvements based on them (e.g., Leaky ReLU, etc.). The mathematical form of Sigmoid function is shown in the following formula:

(1) $$\begin{array}{c} f\left(x\right)=\frac{1}{1+e^{-x}}. \end{array}$$

The Sigmoid function is shown in Figure 2.

The Sigmoid function transforms the continuous real value of the input into the output between 0 and 1. The curve is continuous and smooth. However, since its derivative is also between 0 and 1, the gradient will disappear when the gradient of deep neural network is transmitted back, which makes the network difficult to converge. In addition, the mean output of Sigmoid function is not 0, which will lead to the neuron at the latter layer getting the nonzero mean output of the upper layer as input. As a result, in the process of back-propagation, the weight of the network is updated in two extremes: both are updated in the positive direction or both are updated in the negative direction, resulting in slow convergence. Moreover, the analytic formula of Sigmoid function contains curtain operation, which will consume more time for the computer to solve, while for the large-scale deep neural network, multicurtain operation will consume more training time.

Figure 3 is a schematic diagram of Tanh function.

The Tanh function is the hyperbolic tangent function, derived from the hyperbolic sine and cosine. The formula is shown as follows:

(2) $$\begin{array}{c} f\left(x\right)=\frac{1-e^{-2x}}{1+e^{-2x}}. \end{array}$$

The value range of Tanh function is between (0, 1), and it is an odd function with strict monotonically increasing curve. It has the property of continuous smooth, which further optimizes the Sigmoid function and facilitates the derivation of the model [11]. Compared with Sigmoid function, due to its saturation, it is easy to produce gradient disappearance in neural network back-propagation algorithm, which leads to the problem of difficult training. Moreover, the output distribution of its function value is not zero mean. Therefore, this paper prefers Tanh function, also known as hyperbolic tangent function, when selecting activation function in neural network.

The corresponding image of ReLU function is shown in Figure 4.

As mentioned above, the value of Tanh function is located on (−1, 1), which solves the problem that the mean output value of Sigmoid function is nonzero and the convergence speed is faster. However, it also has problems of gradient disappearance and curtain operation. The most commonly used activation function is ReLU [12]. The ReLU function is a maximization function defined as *f*(*x*) = Max(0, *x*). Since the derivative value of ReLU function is 0 or 1, the problem of gradient disappearance is solved. Moreover, ReLU function only needs to judge whether the input value is greater than 0, so its calculation speed is very fast, and its convergence speed is much faster than those of Sigmoid function and Tanh function. However, the mean output value of ReLU function is not 0, and since the derivative value of ReLU function may be 0, some neurons may never be activated, resulting in the corresponding parameter values never being updated.

### 2.2. Convolutional Neural Network

Convolutional neural networks, CNN, as a deep learning algorithm, are widely used in computer vision, natural language processing, and other fields [13]. The concept of local receptive field is introduced to simulate the construction of biological vision mechanism. Compared with fully connected neural network, convolutional neural network reduces the number of parameters between neurons through weight sharing mechanism, thus reducing the network training time. Convolutional neural network consists of three parts: input layer, hidden layer, and output layer. The input layer can input multidimensional data, and the standardization of data is beneficial to improve the effect of network. Hidden layers mainly include convolution layer, excitation layer, pooling layer, and full connection layer.

  Convolution layer: the task of the convolution layer is to extract the feature vectors of the input data. As the core of the convolutional neural network, the convolution layer contains multiple convolution kernels for convolution operations. Each parameter of the convolution kernel is multiplied and summed up with the corresponding local pixel value to obtain the result of the convolution layer. Then the convolution kernel maps all regions of the input data one by one in the form of a sliding window to obtain the input characteristic information.
  Excitation layer: in the neural network, each neuron node receives the output value of the neuron at the upper layer as the input value of the neuron and transmits the input value to the next layer. The neuron node at the input layer directly transmits the input attribute value to the next layer. In the multilayer neural network, in order to avoid the linear relationship between the output and input of the neuron node, it is necessary to introduce nonlinear function to enhance the expression ability of the network, which is called excitation function (also known as activation function).
  Pooling layer: after feature extraction by the convolutional layer, the input data information can be directly sent into the feature classifier in theory, but it requires a lot of calculation and is prone to overfitting. In order to reduce the magnitude of network parameters and the degree of overfitting of the model, it is necessary to carry out sparse processing on the feature graph and replace the results of a single point in the feature graph with the feature graph statistics of its adjacent areas, namely, pooling/sampling processing.

Convolutional neural network is generally composed of a group of *n* independent filters, which are convolved with images, respectively, to obtain *n* feature maps. For a specific feature map, each neuron is only connected to a small part of the input image, and all neurons have the same connection weight. Another important part of CNN is the pooling layer. This method is used to reduce the spatial size of feature graph and reduce the number of parameters and computational complexity [14]. The most commonly used pooling technique is max pooling, where only the maximum value is extracted from a set of values from a window of size:

(3) $$\begin{array}{c} {\text{Max}}_{i=1,j=1}^{m,n}W\left[i,j\right]. \end{array}$$

The general architecture of CNN is composed of convolution layer, nonlinear function, and max pooling layer. ReLU (rectified linear unit) is the most commonly used nonlinear function and is defined as

(4) $$\begin{array}{c} R\left(z\right)=\text{Max}\left(0,z\right). \end{array}$$

### 2.3. Recurrent Neural Network

Recurrent neural network (RNN) is mainly used to process sequential data, which can mine temporal and semantic information in data [15]. The biggest characteristic of the recurrent neural network is that it can realize the “memory function.” In terms of network structure, the input of the hidden layer at a certain moment includes both the information of the input layer and the output information of the hidden layer at the previous moment, maintaining the dependence between data.

Previously, due to the fact that the convolution of the neural network output only considered the influence of one input without considering the influence of the other input, the convolution through neural network can be a success in the field of computer vision, but, in some situations related to the time order (such as video of the next frame document context and prediction), performance is unsatisfactory, and the neural network can develop cycles [16]. The recurrent neural network not only considers the input of the previous moment but also remembers the previous information and applies it to the calculation of the current output; that is, the nodes between the hidden layer are connected instead of unconnected, and the input of the hidden layer includes not only the output of the input layer but also the output of the hidden layer at the last moment. The working principle of the recurrent neural network is shown in Figure 5.

As shown in Figure 5, the working process of recurrent neural network follows the following steps:

(1) Input *XT* − 1 at *t* − 1 is sent to the network for calculation to obtain the output *OT* − 1 and the hidden layer state *ST* − 1 at *t* – 1.
(2) The same weight matrix is used to calculate the output at each moment; that is, the weight matrix *W* is shared at all moments.
(3) The network continues to receive the input at the next moment until the end of the input sequence.
  (5) $$\begin{array}{c} O_{t}=g\left(V_{S_{t}}\right),\\ S_{t}=f\left(U_{X_{t}}+W_{S_{t-1}}\right). \end{array}$$

Since the recurrent neural network processes sequential data, as shown in formula (6), the second formula can be repeatedly inserted into the first formula to obtain

(6) $$\begin{array}{c} Ot=g\left(V_{S_{t}}\right)\\ =V\left(f\left(U_{X_{t}}+W_{S_{t-1}}\right)\right)\\ =Vf\left(U_{X_{t}}+Wf\left(U_{X_{t-1}}+W\left(f\left(U_{X_{t-1}}+W_{X_{t-1}}\right)\right)\right)\right)\\ =Vf\left(U_{X_{t}}+Wf\left(U_{X_{t-1}}+W\left(f\left(U_{X_{t-1}}+W{\left(U_{X_{t-1}}+\ldots \right)}_{X_{t-1}}\right)\right)\right)\right). \end{array}$$

The commonly used training algorithm of RNN is the Backpropagation Through Time (BPTT) algorithm, which has the same basic principle as BP algorithm and consists of four steps:

1. Calculate the output value of each neuron forward.
2. Reversely calculate error term 6 of each neuron, which is the partial derivative of the weighted input Nety of the error function *E* to neuron *J*.
3. Calculate the gradient of each weight.
4. Finally, the stochastic gradient descent algorithm is used to update the weight.

### 2.4. Related Technologies

In this paper, the neural network model is constructed and trained by using TensorFlow, image information is read by using Open CV, and the front-end page of children's picture reading and speaking system is constructed by using HTML5, CSS, and jQuery, and the server end of the system is built by using Flask framework. The above technologies are described below.

#### 2.4.1. TensorFlow

The model consists of three parts: data model tensor, computational model data flow graph, and operation model session. TensorFlow is versatile and flexible, which can be used in many fields [17].

#### 2.4.2. OpenCV

OpenCV is an open-source image processing software library written in C++ language for computer vision, with C++, Python, Java, and MATLAB interfaces; it is easy to operate and is widely used in object recognition, image segmentation, machine vision, and other tasks [18].

In the process of extracting image features with convolutional neural network, the cv2.imread() function in OpenCV is used to read image information when input image data. The imread() function takes two arguments, the image path and the form in which the image is read.

#### 2.4.3. HTML5, CSS, and jQuery

In recent years, HTML5+CSS + jQuery has become the mainstream method of website front-end responsive layout. The three following technologies are introduced.

*(1) HTML5*. HTML5 (HyperText Markup Language 5) is a language description method for building and presenting Web content [19]. It adds many features to the version of HTML4, such as intelligent forms, drawing canvas, multimedia, geographical positioning, data storage, and multithreading. In terms of code, HTML5 has added many new elements and features to better handle today's Web applications. HTML5 combines a variety of technologies to bring the Web into a mature application platform, allowing programs to run through the Web browser, bringing users a convenient experience.

In the implementation of the system in this paper, the new API Speech Synthesis Utterance in HTML5 is used to express the content of images to children in the way of “speaking,” which meets the basic needs of children to imitate actions. Speech Synthesis Utterance is used to synthesize the specified text into corresponding speech, including configuration items that specify how to interact with children (language, volume, tone, etc.).

*(2) CSS*. CSS (Cascading Style Sheets) is a computer language for not only statically styling Web pages but also dynamically defining elements of a Web page in conjunction with a variety of scripting languages [20]. CSS can define the style structure of page elements, such as font, color, and location. These styles can be stored either directly on an HTML page or as a single style file.

*(3) jQuery*. Before introducing jQuery, you need to understand JavaScript. JavaScript is a dynamic scripting language that is widely used in HTML pages, adding dynamic functions to HTML pages and establishing a real-time, dynamic, and interactive relationship between users and Web pages [21]. AJAX is used to communicate between the browser and the server without refreshing the whole page. The server will no longer return the whole page but will return a small amount of data and update some nodes through JavaScript DOM. During the data transmission, xml, json, and other formats can be adopted. In this system, the data format is json.

#### 2.4.4. Flask

Flask [22] framework is a lightweight Python framework for network development, along with Django, Tornado, and so forth. Flask framework is adopted in this paper. The main objectives are as follows:

1. The Flask framework is lightweight, easy to operate, and easy to develop.
2. The system is small; Flask framework can realize Web service in a short time.
3. Python programming language is used to achieve relevant functions, and image text description model can be called.

Flask assigns a view function to a URL in the application. Whenever the user accesses the URL, the system executes the view function assigned to the URL, retrieves the return value of the function, and displays it in the browser.

#### 2.4.5. Gated Cyclic Unit Neural Network

LSTM has been widely used in the field of natural language processing, but some shortcomings will be exposed in its use, such as too many parameters and too complex internal calculation, which lead to too long training time. A simpler model was further proposed, which combined the unit state and hidden layer state of LSTM and merged the input gate and forgetfulness gate into update gate in the way of synthesis. Meanwhile, cell state and hidden state HT were also combined, which were different from LSTM in the processing of current new information calculation.

In the GRU model, only two gates, one update gate and one reset gate, are left. This method not only retains the relevant effect of LSTM but also simplifies the structure and makes it have better convergence. Compared with LSTM, GRU combines the forgetfulness gate and the input gate into a single update gate and also blends the cell state and the hidden state. GRU model is a very popular variant based on LSTM because it has a simpler structure, fewer parameters, and similar effects compared to LSTM model.

## 3. Research on Simulation Algorithm of Children's Physical Training

### 3.1. Dynamic Image Feature Extraction

RNN network has a very good effect in processing computer motion recognition, because it has the same effect as human eyes in completing image feature processing. With the development of RNN, the research of computer motion direction is also gradually deepened. Computer-aided motion technology belongs to the subclass of computer dynamic direction capture. With the development of RNN, computer motion also develops. The last full connection layer or pooling layer in circulating neural network is one of the feature extraction methods of moving image. The loop layer contains more detailed target information, such as position change and amplitude. Image coding began to use higher level cyclic features to achieve the acquisition of more information from the image. In this paper, the Faster R-RNN network was used to extract the features of each local region of the image [23]. See Figure 6 for the specific model.

It can be seen from Figure 6 that the Faster R-RNN network can be summarized into the three following levels: First, the Faster R-RNN can efficiently generate the region containing the object to be detected accurately by training the RPN network. Secondly, the Faster R-RNN extracts the features of different objects to be detected from the same image cyclic features. The sharing of such image features provides not only spatial information but also accurate regional information and feature information of objects to be detected. Finally, the penultimate layer network of Faster R-RNN was used to extract top-k interesting high-dimensional features.

### 3.2. Dynamic Detector

The pretrained model is fine-tuned. Four categories were used in this paper, among which the classic VGG-16 network was used for motion feature extraction, and the embedding space was set as 2048 dimensions. The results of the dynamic detector on the test set were 86% of hands raised, 79% of legs extended, 85% of limbs, and 89% of fine twisting.

### 3.3. Normative Mechanism of Goal Guidance

When a series of coherent movements are carried out, their complex processes are often ignored by humans, and normative mechanisms emerge. Since the standard mechanism of target guidance is very classic in the study of motion precision task, this paper finally adopts this mechanism as the extraction of precision degree of dynamic picture process.

### 3.4. Nonlinear Layer

In this paper, multiple nonlinear layers of learning are used in the model, which can simulate some transitions of dynamic images. That is, when the motion is input to the cyclic core, the convex linear transformation (affine transformation) can be performed on each small region. After the transformation is completed, a rectified linear unit (ReLU) can be performed. In our implementation, each nonlinear layer is activated using gated hyperbolic tangent.

The implementation function of each layer is *f*_*a*_ : *x* ∈ *R*^*n*×*m*^⟶*y* ∈ *R*^*n*^, where we have the following definitions:

(7) $$\begin{array}{c} \bar{y}=\tanh\left(Wx+b\right),\\ g=\sigma \left(Wx+b\right),\\ y=\bar{y}\circ g, \end{array}$$

∘ is the element multiplication in Hadamard multiplication, *σ* represents the Sigmoid function, *W* ∈ *R*^*n*×*m*^ represents the weight during training, *b* ∈ *R*^*n*^ represents the error of training, and vector *g* is the gating of function $\bar{y}$ using multiplication to obtain the intermediate value.

### 3.5. Joint Embedding of Models

Since the setting standard of dynamic motion dataset is similar to the setting of Image Caption problem, most of the algorithms that rank top of dynamic motion model adopt the processing method similar to this image processing technology. The idea of joint embedding effectively deals with the bottleneck in the field of dynamic image annotation, so many algorithms in the dynamic motion model use this idea. According to the above analysis, the model is constructed based on joint embedding. The joint feature of motion and target is expressed as *q*, and the feature of image $\hat{v}$ connects a Hadamard product, namely, element multiplication, through nonlinear layer:

(8) $$\begin{array}{c} h=fq\left(q\right)\circ fv\left(\hat{v}\right). \end{array}$$

### 3.6. Output Classifiers

In the training of image and language features, the dynamic motion model is regarded as a special classification problem. In the case of image features and target features as inputs, the exact position can be regarded as a unique classification. A set of candidate answers, called the output vocabulary in this paper, are predetermined by all correct answers at the motion positions that occur more than 8 times in the training set. *N* = 3079 candidate answers meet this condition in dynamic motion model V2.0 dataset. In fact, the dynamic motion model can be viewed as a multilabel classification task. Each training task in the dynamic motion model V2.0 dataset is associated with one or more answers. If there is disagreement among human annotators, especially those with ambiguous actions and multiple or synonymous repeated movements, multiple answers and zero-to-one accuracy can occur.

Multilabel classifier data is mainly predicted by feature fusion parameter *h* and linear mapping parameter *W* 0 to predict the score $\hat{s}$.

(9) $$\begin{array}{c} \hat{s}=\arg\;\max\left(W\circ f\circ \left(h\right)\right). \end{array}$$

Generally speaking, logistic regression uses the cross entropy of information and network distribution, and the realization method of the cross-entropy function depends on the realization method of the answer. Choose to use soft target scores. The last step is logistic regression to prejudge the accuracy of each moving node. The target loss function is shown in formulas (3), (4), and (6)–(10):

(10) $$\begin{array}{c} L=-\sum_{i}^{M}\sum_{j}^{N}s_{ij}\log\left({\hat{s}}_{ij}\right)-\left(1-s_{ij}\right)\text{log}\left(1-{\hat{s}}_{ij}\right), \end{array}$$

where *M* represents the number of training questions, *N* represents the number of candidate answers, index *i* is executed on *M* training questions, and index *j* is executed on *N* candidate answers. *S* stands for the soft accuracy of the correct answer.

## 4. Test Process and Result Analysis

The purpose of this experiment is to verify that the proposed simulation system is able to judge the accuracy of children's movement in both natural and real-time ways. In addition, it can also be proved that the framework model of training mentioned above can well meet the movement requirements in customized scenarios.

### 4.1. Test Environment

In the training of network model, complex and huge matrix operation is needed. In recent years, with the rapid development and continuous update of CPU, it is suitable for intensive floating point operation with high efficiency, making the learning process of artificial intelligence network model faster and gradually realizing the requirements that cannot be reached by the original CPU. Because the test in this paper has a large number of datasets, the operating environment is required. The specific test environment is shown in Table 1.

### 4.2. Introduction to Evaluation Criteria

This experiment uses the 2.0 abstract image dataset under the dynamic motion model and the 10K synthetic scene dataset. In the 2.0 abstract image data set, all nodes are collected manually to ensure the accuracy of the dataset. Therefore, a new evaluation index was introduced.

### 4.3. Test Setup

In the category of possible motion images, the corresponding action nodes can be divided into four types: TrueM-TrueAns, where there is one correct action node but the rest of the actions are irregular; FalseM-TrueAns, where there is one false action but the rest of the actions are correct; FalseM-FalseAns, where all are entirely incorrect; and TrueM-FalseAns, where all are exactly correct.

During testing, input dynamic images, moving nodes, and target labels. If the model manages to output the exact answer in the right way, it is considered the correct action. Performance depends on the accuracy of the model. In this paper, clipart dataset of balanced dataset in dynamic target model V2 is used, and precise target label is added in the preprocessing of dataset. For each of the possible 4 predictive action node tags, the motion features are calculated, and then the problem features and target tags are passed to the gated loop unit neural network as inputs to generate feedback of motion accuracy. If the feedback on the image is hitting the target point, then all the movements are correct throughout the movement.

### 4.4. Show the Effect Drawing

The experimental output samples are given, and the typical outputs covering four basic movements are given. Six motion categories were used in the study, and Figure 7 shows the sample results selected from the model in this article.

The results showed the relevant exercise categories and the judgment of exercise results. These actions are very easy to distinguish, and the judgment criteria given are very clear, so as to achieve the correlation between children's motor input and target output. The sample results verify that children can completely use this system to simulate sports scenes, and the training simulator can judge whether these series of actions meet expectations according to several special nodes of children's action amplitude and regard the actions that meet expectations as correct; otherwise, they will be regarded as having problems. The results of the model test show that the design of the simulation system is reasonable and the accuracy can meet the requirements of children's normal sports.

### 4.5. Analysis and Comparison with Other Models

#### 4.5.1. Model Performance Analysis

Although the target detector has a good performance in the test set, this effect must be verified by the size of the fit degree in the target matching model. This performance depends on how high the TrueM-TrueAns metric can be.  Table 2 shows the overall percentage of motion output.

It can be seen from Table 2 that, in FalseM-TrueAns, the conventional part of target matching in the modified network model is slightly higher than that in the traditional neural network model, but, in FalseM-FalseAns, the accuracies of action process output and target output in the modified network model are slightly lower than those in the traditional neural network model. These two categories account for a certain percentage and are directly affected by the propagation effect of the emotion detector in the dynamic image, thus affecting the overall performance of the model. In TrueM-FalseAns class, the target node part of the present model is almost the same as the traditional model, which is only affected by the basic functions of the dynamic love image model. The addition of the improved process object tag does not affect the basic performance of the dynamic image model. To sum up, the network of dynamic image model needs to be modified accordingly. The process target detector is added to the RNN + LSTM model. The first improved model adopts pretrained FTP-RNN, as well as the second improved image features extracted by target matching mechanism, so that RNN + LSTM can directly extract global image features and increase the chance of error rate extraction.

#### 4.5.2. Model Comparison

Table 3 shows the data for comparing this model with other models.

The proportion consistency of precision comparison results between models in Table 3 shows that the addition of process target detection in the model network in this paper does not significantly interfere with the final evaluation results but, on the contrary, enables the dynamic image model to carry out richer analysis and understanding of image features. The final action node is not primarily used for the identification task of the correct action. Even after the dataset was trimmed, many images in the dataset were classified as invalid because they were not captured to the node, which is partly responsible for this phenomenon. In some cases, the overall performance of the dynamic image recognition model presented in this paper is slightly better than that presented in the literature, which is due to the target matching mechanism guided by process and result targets adopted in this model. Process nodes and final nodes are fused together as a problem to enhance the attention of the image process. Compared with the earlier traditional neural network model, multimodal residual learning, and LSTM + RNN, the improved RNN model in this paper is also in a leading position.

## 5. Conclusion

This paper introduces the development of website education in today's era, expounds its research significance, and puts forward the existing online education platform with artificial intelligence and virtual reality technology ideas and framework. The improved neural network in artificial intelligence technology and Web3D in virtual reality technology are introduced, respectively.

On this basis, this paper puts forward an algorithm for children's physical training simulation system. This paper fully investigated and integrated ideas and finally selected the abstract dataset on dynamic image processing V2. Through the corresponding design objectives, 10K pictures with 3D synthetic children's sports training dataset were made to build the network of this paper. The network adopts the method of joint embedding, which encodes the image, text, and action nodes, respectively, to project them to a common dynamic space and carries out feature fusion.

Finally, a simulation system algorithm for children's physical training is constructed. Through the comparison experiment with the traditional neural network algorithm, the existing simulation system design ideas are comprehensively compared, and its advantages and disadvantages are explored. The modular development framework is formed through several times of modifying the algorithm model. Finally, the accuracy of the algorithm system in this paper is significantly higher than that of the traditional neural network model without improvement. The human-computer interaction system of children's physical training under Web3D environment is completely constructed.

## Figures and Tables

**Figure 1:** Schematic diagram of neurons.

**Figure 2:** Sigmoid transfer function.

**Figure 3:** Tanh function.

**Figure 4:** ReLU function.

**Figure 5:** Recurrent neural network.

**Figure 6:** Processing process of the Faster R-RNN algorithm.

**Figure 7:** Test output sample.

**Table 1:** Test environment setting.

Name	Parameter
Operating system	64-bit Ubuntu 18.04
Graphics processing unit (GPU)	GeForce GTX 1080Ti
Memory/hard disk capacity	64 G/2 T
Programming environment	PyTorch Pyhton 3.6

**Table 2:** The model's overall percentage of answers in each category (%).

Model	Classification			
	TrueM-TrueAns	FalseM-TrueAns	FalseM-FalseAns	TrueM-FalseAns
CNN + LSTM + M	52.7	9.2	20.9	17.2
The model in this paper	54.9	12.3	16.3	17.5

**Table 3:** Data for comparison between the model in this paper and other models (%).

Model	Yes/no	Num.	Other	All
Multimodal residual learning	77.79	47.98	48.90	61.89
LSTM + CNN	76.25	49.26	55.06	63.32
BUTD	79.01	52.03	61.05	68.91
The model in this paper	78.98	51.97	61.19	69.03

## Data Availability

The dataset can be accessed upon request.
